This article has been retracted.

# A Short Caspase-3 Isoform Inhibits Chemotherapy-Induced Apoptosis by Blocking Apoptosome Assembly

**DOI:** 10.1371/journal.pone.0029058

**Published:** 2011-12-22

**Authors:** Frédérique Végran, Romain Boidot, Eric Solary, Sarab Lizard-Nacol

**Affiliations:** 1 Unit of Molecular Biology - Centre Georges François Leclerc, Dijon, France; 2 Federative Institute of Research IFR “Santé-STIC” - University of Burgundy, Dijon, France; 3 UMR-INSERM U-866, Dijon, France; University of Hong Kong, Hong Kong

## Abstract

Alternative splicing of caspase-3 produces a short isoform caspase-3s that antagonizes caspase-3 apoptotic activity. However, the mechanism of apoptosis inhibition by caspase-3s remains unknown. Here we show that exogenous caspase-3 sensitizes MCF-7 and HBL100 breast cancers cells to chemotherapeutic treatments such as etoposide and methotrexate whereas co-transfection with caspase-3s strongly inhibits etoposide and methotrexate-induced apoptosis underlying thus the anti-apoptotic role of caspase-3s. In caspase-3 transfected cells, lamin-A and α-fodrin were cleaved when caspase-3 was activated by etoposide or methotrexate. When caspase-3s was co-transfected, this cleavage was strongly reduced. Depletion of caspase-3 by RNA interference in HBL100 containing endogenous caspase-3s caused reduction in etoposide and methotrexate-induced apoptosis, whereas the depletion of caspase-3s sensitized cells to chemotherapy. In the presence of caspase-3s, a lack of interaction between caspase-3 and caspase-9 was observed. Immunoprecipitation assays showed that caspase-3s binds the pro-forms of caspase-3. This result suggested that the absence of interaction with caspase-9 when both variants of caspase-3 are present contribute to block the apoptosome assembly and inhibit apoptosis. These data support that caspases-3s negatively interferes with caspase-3 activation and apoptosis in breast cancer, and that it can play key roles in the modulation of response to chemotherapeutic treatments.

## Introduction

Caspases are a family of evolutionary conserved cysteine proteases that play a central role in a majority of apoptotic cell death pathways. Death signals activate the proteolytic cascade of caspases through two main pathways, i.e. an extrinsic pathway that starts at the level of plasma membrane death receptors and an intrinsic pathway that activation is a response to irreversible cellular damage [1]. Both pathways converge to the activation of caspase-3, the closer homolog of the in *Caenorhabditis elegans* CED-3 [2]. Procaspase-3 is a 32 kDa caspase-3 zymogen (also known as CPP32). CPP32 exists in the cells as inactive dimmers. Its proteolytic cleavage on C-terminal side of aspartate residues eliminates the pro-domain, separates the remaining protein into a large and a small subunit and generates an active tetramer constituted by two large and two small subunits. In turn, caspase-3 activates downstream enzymes of the caspase family and contributes with them to generate the characteristic apoptotic cell death phenotype.

Activation of caspase-3 is required for membrane bleeding and internucleosomal DNA fragmentation that occur during apoptosis. Caspase activity is regulated at several levels, including gene transcription and post-translational modifications. The alternative splicing of *caspase* genes generates full-length and truncated proteins whose functions can be antagonistic [3]. This characteristic maintains the threshold of response to certain levels of stimuli [4].

The human *Caspase-3* gene is located on 4q33-q35.1 and possesses 2635 base pairs leading to 7 exons. Its alternative splicing generates two transcripts, caspase-3 and caspase-3s that were detected in all the studied tissues [5] and may have different apoptotic activities [5], [6]. The principal mRNA variant, caspase-3, is 834 base-long and the short transcript, caspase-3s, has lost the sixth exon leading to a loss of 122 bases (representing 95 amino-acids initially present in the procaspase-3 protein). The lost sequence includes the short subunit and the C-terminal part of the long subunit in which is located the QACRG motif that participates in the formation of the catalytic site. The caspase-3s protein has around a 20 KDa molecular weight and expression of the short isoform of caspase-3 in 293T cells prevents DNA fragmentation and poly(ADP-ribose) polymerase 1 (PARP1) cleavage in response to an apoptotic stimulus [5].

The role of caspase-3 in the response of breast cancer cells to chemotherapeutic drugs remains a controversial issue. The lost of caspase-3 expression as well as defaults in cytochrome c release from the mitochondria, which is requested in most apoptotic pathways to activate caspase-3 through caspase-9 activation, are associated with multidrug resistance. Accordingly, expression of caspase-3 in the human MCF-7 breast tumor cell line (which is deficient for caspase-3) restores the apoptotic response to the topoisomerase II inhibitor, etoposide [7]–[9]. Caspase-3 was also involved in breast cancer cell apoptosis upon exposure to anthracyclines [9]–[12] and cisplatin [13]–[16]. Its role in tumor cell response to paclitaxel has been challenged [17]–[24].

Currently, the role of caspase-3s in chemotherapy response is unexplored. We also previously studied the impact of caspase-3s expression in a population of breast carcinomas treated with neoadjuvant cyclophosphamide-based chemotherapy and observed an inverse relationship between caspase-3s/caspase-3 ratio level expression and pathological response [6]. Therefore, the present study was performed to precise the molecular mechanism in apoptosis inhibition of caspase-3s by using breast tumor cell lines MCF-7 treated by various chemotherapeutic agents known to induce an apoptotic mode of cell death.

## Materials and Methods

### Cell lines

Human breast cancer cell lines MCF-7 (deficient for caspase-3), HBL-100 and MDA-MB-231 (proficient for caspase-3) were purchased from the ATCC (American Type Culture Collection, Manassas, VA, USA). The cell lines were cultured according to the manufacturer's instructions.

### Full-length cDNA synthesis and cloning

The full-length of caspase-3 and caspase-3s coding sequences were obtained using SuperScript™ One-Step long templates RT-PCR (Invitrogen, Carlsbad, CA, USA) with 1.25 µg of total RNA from the UACC3199 cell line (Arizona Cancer Center Tissue Culture Shared Resource) containing high levels of the two transcripts. Specific primers used were reported in Table S1. PCR program was performed by one cycle at 45°C for 30 min, 94°C for 2 min followed by 35 cycles of 15 s at 94°C, 30 s at 50°C, 1 min at 68°C, and one final cycle for 5 min at 72°C (Abi Prism 9700 thermocycler, Applied Biosystems, Foster City, CA, USA). The two transcripts were separated by a 3% agarose gel electrophoresis and purified by specific extraction with QIAquick Gel Extraction Kit (Qiagen, Courtaboeuf, France).

The inserts were cloned into pcDNA3.1/CT-GFP-TOPO or pcDNA3.1/CT-YFP-TOPO and amplified in One Shot® TOP10 Chemically Competent E. Coli with Fusion TOPO® TA Expression Kits (Invitrogen). The plasmids from a few randomly picked colonies were isolated. The orientations of the caspase-3 or caspase-3s fragments were tested by PCR and automatic sequencing as described below.

### Stable transfection

For stable transfection, 5×10^5^ MCF-7 and HBL100 cells were grown in a medium without antibiotics in 12-well plates. Two days later, cells were transfected with 0.5 µg of plasmid containing either caspase-3 or caspase-3s insert and with GFP or YFP control vector. Stable transfections were performed by LipofectAMINE 2000 (Invitrogen) according to manufacturer's instructions. The stable colonies were selected by 1000 µg/ml Geneticin® or 10 µg/ml Blasticidin (Invitrogen). To ensure that the inserts were sufficiently expressed, the transfection efficiency was controlled by quantitative real-time RT-PCR amplification, the presence of GFP and YFP was controlled by microscopy and the presence of extrinsic caspase-3 and caspase-3s was determined by Western Blot. Relative change expressions were calculated between control and transfected cells.

### Caspase-3 and caspase-3s extinction by siRNA

HBL100 or MDA-MB-231 cells (3×10^4^ per wells), which are proficient for caspase-3, were grown in a medium without antibiotics in 6-well plates during 2 days. Transfections (procaspase-3 siRNA: CGACUUCUUGUAUGCAUACUCCACA, caspase-3s siRNA: GGGTTATTATTCTTGGCGAA) were performed by LipofectAMINE 2000. Twenty four, 48, 72 and 96 hours of extinction were tested by Western Blot (Figure S2A) or quantitative PCR (Figure S2B). Cytotoxic treatments were performed during the best extinction time lapse (Figure S2A and B). For treatment after caspase-3s down-regulation, chemotherapeutic drug yields were 10 fold inferior to the IC50.

### Sequencing of PCR products

The specificity of all PCR amplifications was verified by sequencing of PCR-products. Briefly, products were excised from 3% agarose gels and isolated as described above. The purified PCR products were sequenced using the Abi-Prism Big Dye Terminator Cycle Sequencing Ready Reaction Kit (Applied Biosystems) with the respective primers used in the initial PCR according to the manufacturer's protocol.

### RNA extraction, cDNA synthesis, and Quantitative real-time PCR amplification

Total RNA was extracted with Trizol reagent (Invitrogen) and its quality was checked by 28S/18S ratio on agarose gel. One microgram of total RNA was reverse transcribed as previously described [6].

For real-time PCR, amplification was performed in a total volume of 25 µL in the presence of 600 nM of each primers, 200 nM of probe, 12.5 µL of Universal Master Mix (Applied Biosystems), and 12 ng of cDNA (or water as negative control). PCR was performed with an initial denaturation step of 10 min at 95°C, followed by 40 cycles of 15 s at 95°C and 1 min at 60°C. All samples were amplified in duplicate and results were analyzed at the C_T_ level. Control 18S reactions (Applied Biosystems) were used to normalize ΔC_T_ values.

### Total protein extractions

Total protein extraction was performed by addition of lysis buffer (20 mM Tris pH 7.5, 150 mM NaCl, 1 mM EDTA, 1 mM EGTA, 1% Triton X-100, 2.5 mM Sodium pyrophosphate, 1 mM β-Glycerophosphate, 1 mM Na_3_VO_4_, 1 µg/ml Leupeptin, 1 mM PMSF added immediately prior to use) on cell monolayer for 5 min on ice. Afterwards, the lysate was harvested and sonicated.

### Western Blot analysis

30 µg of protein extracts were separated SDS-PAGE 10% acrylamide and transferred to PVDF or nitrocellulose membranes (according to the molecular weight of the protein) with an electrophoretic transfer apparatus. After blocking with buffer containing 3% of ECL Advance™ blocking agent (GE Healthcare, Buckinghamshire UK) in PBS/Tween 0.3% for 1.5 hour at room temperature, the membrane was probed with specific polyclonal antibodies (Abcam, Cambridge, UK) diluted in blocking solution (β-actin 1/25000, caspase-3 1/7500, GFP 1/50000, caspase-9 1/1000, APAF-1 1/1000, lamin A 1/4000, or α-fodrin 1/2000) for 1 hour at room temperature. The antibody used for procaspase-3 and caspase-3 detection was generated with the epitope residues between amino acids 161 and 175. This part of the protein is common to procaspase-3 and caspase-3 as it is located in the large subunit.

The GFP antibody recognizes YFP in YFP transfected cells and thus the caspase-3s YFP tag. Next, the membrane was incubated with biotinylated anti-rabbit IgG (1∶50000 in blocking solution) secondary antibody (Invitrogen) 30 min at room temperature. Then, the membrane was probed with streptavidin-HRP (1/50000) for 15 min at room temperature in PBS/Tween 0.3%. Signals were detected using a chemiluminescent detection system (ECL Advance™ Western Blotting Detection Kit; GE Healthcare) and Chemidoc XSR device (Bio-Rad).

### Flow cytometric assessment of apoptosis after dual staining with Annexin-V-PE and 7AAD

Apoptosis was induced by a large scale of chemotherapeutic drugs in the two cell lines (MCF-7 and HBL100) (Table S2). Assessment of apoptosis was accomplished by measuring Annexin-V-PE and 7AAD staining (Apoptosis Detection Kit I BD Pharmingen™, Franklin Lakes (NJ), USA) according to manufacturer's instructions. Cells (30 000) were counted by flow cytometry using Becton Dickinson LSRII and the experiments were performed in triplicate in two different clones.

### Immunoprecipitation assays (IP)

IP assays were carried out on total protein extract of HBL100 cell line with Exacta Cruz matrix (Tebu-bio, Le Perray En Yvelines, France) according to manufacturer's instructions and analyzed by western blot.

### Fluorescence microscopy

Wild-type, non tagged procaspase-3 or caspase-3s stably transfected MCF-7 cells were transiently transfected with procaspase-3-GFP or caspase-3s-YFP. Cells were plated onto 6-well plates for 24 hours, then treated or not with anticancer drugs for indicated times before replacing the culture medium with phenol red-free medium. Cells were scanned in phase contrast, and with a GFP or YFP filter under UV light.

### Statistical analysis

Data were analyzed using the student t test on the Statview 5.0 software.

## Results

### Caspase-3s inhibits drug-induced apoptosis in breast cancer cells

We previously showed that in breast carcinoma, increase in caspase-3s/caspase3 ratio expression was significantly associated with chemoresistance to cyclophosphamide-based neoadjuvant treatment [6]. To go further, procaspase-3 and caspase-3s were stably transfected, either alone or in combination in MCF-7 cells. The constructs were fused to GFP (pro-caspase-3) or YFP (caspase-3s) and the GFP vector was used as a control (Figure S1). Transfected MCF-7 cells were exposed to the topoisomerase II inhibitor etoposide, the tubulin poison vinblastine and the folate metabolism inhibitor methotrexate for 48 hours before analyzing apoptosis induction by the use of a flow cytometry assay. Expression of procaspase-3 cDNA strongly increased the ability of MCF-7 to undergo apoptosis in response to etoposide and methotrexate but did not demonstrate any significant effect on vinblastine-induced cell death in the tested conditions or slightly enhanced their apoptotic response to some of the drugs used (Figure 1A, light grey bars). Expression of the caspase-3s either did not sensitize the cells to drug-induced apoptosis (Figure 1A, black bars). Remarkably, co-expression of both procaspase-3 and caspase-3s completely suppressed the ability of procaspase-3 expression to sensitize MCF-7 cells to etoposide and methotrexate-induced cell death (Figure 1A, dark grey bars). These results were further completed by studying the consequences of caspase-3s and/or procaspase-3 expression on apoptosis induced by a series of other cytotoxic agents in MCF-7 and HBL100 cells. Both cell lines demonstrated specific profiles of sensitivity to drug-induced apoptosis. While procaspase-3 expression (in MCF-7) or overexpression (in HBL100) increased their apoptotic response to cytotoxic agents (5FU, Bleomycin, Cisplatine, Epirubicin, Vincristine or Staurosporine), expression of caspase-3s always counteracted this sensitization (Table S3). Moreover, siRNA experiments targeting a sequence located in the caspase-3 specific exon 6 or a specific sequence of caspase-3s, to down-regulate the expression of procaspase-3 or caspase-3s respectively, in HBL100 cells were performed to determine the effect of endogenous caspase-3s after apoptosis induction. Cells were treated with etoposide, vinblastine and methotrexate for 48 hours. In absence of procaspase-3 (Figure 1B), HBL100 cells were less sensitive to apoptosis induced by etoposide and methotrexate. As expected, in absence of caspase-3s (Figure 1C), both HBL100 and MDA-MB-231 cells were more sensitive to etoposide and methotrexate induced apoptosis, confirming that endogenous caspase-3s plays an important role in caspase-3 dependant apoptosis regulation.

**Figure 1:** Caspase-3s inhibits drug-induced apoptosis. **A.** MCF-7 cells were stably transfected with GFP vector (white), procaspase-3-GFP (light grey), caspase-3s-YFP (black) or with C3-GFP and C3s-YFP (dark grey) and treated with etoposide, vinblastine or methotrexate for 48 H. **B.** HBL100 WT cells (white) were transfected either with scRNA (grey) or with siRNA against procaspase-3 (black). The efficiency of procaspase-3 extinction is shown in the small inset. Apoptosis was next induced by etoposide, vinblastine or methotrexate and detected by flow cytometry. Asterisks correspond to *p*<0.01. **C.** HBL100 and MDA-MB-231 cells (white) were transfected either with scRNA (white) or with siRNA against caspase-3s (black). The efficiency of caspase-3s extinction is shown in the small inset. Apoptosis was next induced by etoposide, vinblastine or methotrexate and detected by flow cytometry. The drug used yields in panel C were 10 fold inferior than the IC50 used in panel B, explaining the differences between controls of panels B and C. Asterisks correspond to *p*<0.01.

### Caspase-3s prevents procaspase-3 activation

We first analyzed procaspase-3 activation in treated MCF-7 cells transfected with pro-caspase-3-GFP or with caspase-3s-YFP. Whereas vinblastine did not demonstrate any effect on procaspase-3 activation (Figure 2A, fifth and sixth tracks), exposure to etoposide and methotrexate induced the proteolytic cleavage of the procaspase-3-GFP into a p40 fragment indicating the activation of caspase-3-GFP (Figure 2A, third and seventh tracks). The expression of caspase-3s-YFP with caspase-3-GFP prevented the ability of etoposide and methotrexate to trigger the proteolytic cleavage of the proenzyme (Figure 2A, fourth and eighth tracks). In procaspase-3 proficient cells, etoposide and methotrexate induced the cleavage of caspase-3 specific substrates, the 70 KDa Lamin-A into a 28 KDa fragment and the cleavage of the 250 kDa α-Fodrin into a 160 kDa fragment [25], [26]. These cleavages were not observed in MCF-7 cells expressing only caspase-3s and in those expressing both procaspase-3 and caspase-3s in response to etoposide (Figure 2B) and methotrexate (Figure 2D). Vinblastine treatment had not effect on Lamin-A and α-Fodrin cleavage (Figure 2C) whatever the pro-caspase-3 or caspase-3s expression.

**Figure 2:** Caspase-3s prevents procaspase-3 activation. **A.** MCF-7 cells stably transfected with caspase-3 were treated with etoposide, vinblastine or methotrexate (lanes 1, 3, 5 and 7). Caspase-3 was cleaved in procaspase-3 transfected cells after 48 hour treatment with etoposide, or methotrexate but not after vinblastine treatment. In procaspase-3-GFP/C3s-YFP co-transfected treated MCF-7 cells (lanes 2, 4, 6, and 8), procaspase-3 cleavage was completely abolished. β-actin was used as loading control. **B–D.** Analysis of lamin-A and α-fodrin cleavage by Western Blot. GFP MCF-7 cells, procaspase-3-GFP (ProC3-GFP) or caspase-3s-YFP (C3s-YFP) transfected cells were treated with etoposide (**B**), vinblastine (**C**) or Methotrexate (**D**) during 48 hours. Lamin-A and α-fodrin were cleaved only in single procaspase-3-GFP transfected cells treated with etoposide or Methotrexate. ProC3-GFP/C3s-YFP co-transfected cells treated with etoposide or methotrexate did not show cleavage of neither lamin-A nor α-fodrin. In accordance with panel A, vinblastine did not induce cleavage of neither lamin-A nor α-fodrin β-actin was used as loading control.

### Caspase-3s influences procaspase-3 location

Fluorescent microscopy analyses of MCF-7 cells indicated that, in the absence of any treatment, procaspase-3-GFP was located mainly in the cytoplasm (Figure 3A, first line), whereas caspase-3s-YFP was in both nucleus and cytoplasm (Figure 3B, first line). Upon exposure to etoposide or methotrexate for 10 hours, part of the GFP-tagged caspase-3 was translocated into the nucleus (Figure 3A, second and fourth lines). After vinblastine exposure, GFP-tagged procaspase-3 remained in the cytoplasm (Figure 3A, third line). Caspase-3s location was not influenced by any treatment (Figure 3B, second, third and fourth lines). When non tagged caspase-3s was stably expressed in MCF-7 cells before transient expression of GFP-tagged procaspase-3, the fluorescent procaspase-3 was located in both nucleus and cytoplasm and exposure to the tested drugs did not change this subcellular repartition (Figure 3C). As expected, when non tagged procaspase-3 was stably expressed in MCF-7 cells before transient expression of YFP-tagged caspase-3s, the fluorescent caspase-3s was located in both nucleus and cytoplasm and again, exposure to the tested drugs did not change significantly this subcellular repartition (Figure 3D). The fluorescent nuclear staining quantification is shown in Table S4.

**Figure 3:** Caspase-3s influences the localization of procaspase-3. Twenty-four hours after GFP-coupled procaspase-3 (C3-GFP) or YFP-coupled caspase-3s (C3s-YFP) transfection in parental MCF-7 cells (**A** and **B** respectively) or in non tagged caspase-3s (C3s) or procaspase-3 (C3) stably transfected MCF-7 cells (**C** and **D** respectively) MCF-7 cells were treated or not with etoposide, vinblastine or methotrexate for 10 hours. Cells were scanned in phase contrast and with a GFP or YFP filter under UV light. Nuclei were delimited by dotted lines. The nulear staining quantification is presented in Table S4.

### Caspase-3s structure predicts an absence of catalytic activity

To understand why caspase-3s has no catalytic activity, we studied its protein sequence and structure. As shown in Figure 4A, caspase-3s has no catalytic site compared with procaspase-3, and especially the cysteine residue that is crucial for the catalytic activity of caspases. Moreover, caspase-3s does not possess the cleavage site between the small and the large subunit, resulting in an absence of cleavage into two subunits. Finally, in the caspase-3s, there are no sites for binding of caspase inhibitors such as Ac-DEVD-CHO [27], XIAP [28]… However, caspase-3s possesses the same pro-domain as procaspase-3, but, contrary to procaspase-3, caspase-3s pro-domain is not cleaved. Indeed, the activation of procaspase-3 is sequential. The first step is the cleavage between the large and the small subunits. Once this cleavage is done, the large+small subunit complex induces the cleavage of the pro-domain, involving the activation of caspase-3. Thus, if the protein is not divided in two subunits, the pro-domain can not be cleaved. Therefore, the absence of caspase-3s pro-domain cleavage may be explained by the absence of caspase-3s cleavage in two subunits.

**Figure 4:** Protein sequence and 3D structure of procaspase-3 and caspase-3s. **A.** Alignment of procaspase-3 (C3) and caspase-3s (C3s) amino acid sequences. Prodomain is framed, amino acids forming the catalytic site are in bold blue, interaction sites with caspase-3 inhibitors are in bold green [27]–[28], cleavage site between small and large subunits are in bold and underlined [28], aspartate residue cleaved during activation are in bold red [29]. **B.** 3D structure of procaspase-3 and caspase-3s. Bold arrows represent the end of common sequence between both proteins and pink asterisks show the β-sheets and α-helixes present in procaspase-3 and absent in caspase-3s.

The difference between pro-caspase-3 and caspase-3s sequences has a strong impact on the 3D structure. In fact, when the pro-caspase-3 3D structure was compared with the caspase-3s one, it appeared that caspase-3s lacked 2 β-sheets and 2 α-helixes compared with procaspase-3 (Figure 4B). These structures are necessary for the catalytic activity of caspase-3.

### Caspase-3s interacts with procaspase-3 and prevents its interaction with apoptosome

To understand the apoptosis inhibition mechanism of caspase-3s, co-immunoprecipitation experiments were performed in HBL100 cells stably transfected with YFP-coupled caspase-3s. Using an anti-caspase-3 monoclonal antibody that targets an epitope located in the short subunit of caspase-3, detecting only procaspase-3 and active caspase-3 but not caspase-3s, we observed, upon exposure to etoposide and methotrexate, caspase-3s interacted with procaspase-3 (Figure 5A). Moreover, co-immunoprecipitation experiments with an anti-GFP antibody (that recognizes caspase-3s tag) demonstrated that, in cells exposed to etoposide or methotrexate, caspase-3s-YFP could pull down procaspase-3 (Figure 5B).

**Figure 5:** Caspase-3s interacts with procaspase-3 and inhibits the apoptosome assembly. **A–B.** This experiment was carried out in HBL100 cells stably transfected with caspase-3s-YFP or YFP alone and treated with etoposide, vinblastine or methotrexate for 48 hours. **A.** In YFP transfected cells, immunoprecipitations were performed with anti-caspase-3 antibody and western blot with anti-GFP (that recognizes YFP in YFP transfected cells and the caspase-3s YFP tag) and anti-caspase-3 antibodies. The results revealed no interaction between caspase-3 and YFP with or without treatment. In HBL100 transfected with caspase-3s-YFP, an interaction between procaspase-3 and caspase-3s after etoposide or methotrexate treatments was observed. **B.** In YFP transfected cells, immunoprecipitations were performed with anti-GFP antibody and western blot with anti-caspase-3 and anti-GFP antibodies. The results revealed no interaction between YFP and procaspase-3 whatever the conditions. In caspase-3s-YFP transfected HBL100, an interaction between caspase-3s and procaspase-3 was observed after etoposide or methotrexate treatment. **C–F.** MCF-7 cells were transfected with empty-vector (YFP), procaspase-3 (ProC3) or caspase-3s-YFP (C3s-YFP) or both caspase-3s-YFP and procaspase-3. The cells were treated or not with etoposide. **C.** Immunoprecipitations were performed with anti-active caspase-9 antibody and western blot with anti-active caspase-9, anti-Apaf-1, anti-caspase3 and anti-GFP (that recognizes caspase-3s tag) antibodies. The results showed that procaspase-3 and caspase-3s interacted, in treated cells, with active caspase-9 and anti-Apaf-1 only when they are alone. As soon as caspase-3s and procaspase-3 are present at the same time, the interaction with active caspase-9 and anti-Apaf-1 was abolished. **D.** Immunoprecipitations were performed with anti-caspase-3 antibody and western blot with anti-caspase-3, anti-Apaf-1, and anti-active caspase-9 antibodies. The results showed that procaspase-3 interacted with active caspase-9 and anti-Apaf-1 in treated cells only in absence of caspase-3s. **E.** Immunoprecipitations were performed with anti-GFP antibody and western blot with anti-GFP, anti-Apaf-1 and anti-active caspase-9 antibodies. The results showed that YFP did not interact with active caspase-9 and anti-Apaf-1 whereas caspase-3s interacted with active caspase-9 and anti-Apaf-1 in treated cells only in absence of procaspase-3. **F.** Immunoprecipitations were performed with anti-Apaf-1 antibody and western blot with anti-Apaf-1, anti-active caspase-9, anti-caspase-3 and anti-GFP antibodies. The results showed that procaspase-3 and caspase-3s interacted, in treated cells, with active Apaf-1 and caspase-9 only when they are alone. As soon as caspase-3s and procaspase-3 are present at the same time, the interaction with Apaf-1 and active caspase-9 was abrogated.

Then, we wondered whether the interaction of caspase-3s with procaspase-3 prevents pro-caspase-3 activation by inhibiting apoptosome assembly. For that, MCF-7 cells were transfected with a vector encoding either YFP alone or the YFP-tagged caspase-3s or procaspase-3 without any tag. These cells were left untreated or treated with etoposide for 48 hours. Afterwards, cell lysates were immunoprecipitated with an anti-active caspase-9 antibody and Apaf-1 antibody representing the Apaf-1/cytochrome c/caspase-9 complex, precursor of apoptosome. The active form of caspase-9 was detected by immunoblot analysis in etoposide treated cells (Figure 5C, Active caspase-9 panel) and its interaction with Apaf-1 was confirmed in etoposide treated samples (Figure 5C, APAF-1 panel). The results showed an interaction between active caspase-9/Apaf-1 and procaspase-3 (as detected with an anti-procaspase-3 antibody) or caspase-3s (as detected with an anti-GFP antibody, recognizing caspase-3s tag) when these proteins were expressed alone in etoposide-treated cells. These interactions were no more detected when both procaspase-3 and caspase-3s were expressed simultaneously (Figure 5C, Procaspase-3 and C3s-YFP panels). The results were confirmed by inverse immunoprecipitation with an anti-procaspase-3 antibody (Figure 5D), an anti-GFP antibody (Figure 5E), and an anti-Apaf-1 antibody (Figure 5F). These results suggested that caspase-3s prevent the apoptosome assembly by sequestrating procaspase-3.

## Discussion

A variety of mechanisms has been described to account for the resistance of breast cancer cells as well as other tumor types to anticancer agents. Indeed, patients often develop drug resistance towards drugs of unrelated structures and activities. To fight against chemotherapy, cancer cells are able to develop various mechanisms of resistance such as activation of survival pathways or apoptosis resistance. Apoptosis resistance can reflect resistance to chemotherapeutic treatments [1]. Caspase-3 is a major pro-apoptotic protein and is a key enzyme in drug-induced apoptosis of tumor cells [9]. In contrast, caspase-3s overexpression in breast carcinomas might be indicative of chemoresistance to neoadjuvant cyclophosphamide-containing treatment [6]. Thus, it was suggested that caspase-3s might be an apoptosis protagonist which could be a new predictive marker of apoptosis resistance. To evaluate this hypothesis, the ability of caspase-3s to counteract apoptosis induced by various pro-apoptotic chemotherapeutic drugs was evaluated in this study with the use of breast tumor cell lines which are deficient or proficient for caspase-3.

The present study demonstrates that caspase-3s, generated by alternative splicing of caspase-3 pre-mRNA, negatively interferes with caspase-3 activation and apoptosis in breast cancer cells exposed to cytotoxic drugs. This effect appears to involve an interaction of caspase-3s with procaspase-3 that prevents its recruitment in the apoptosome and its activation.

Our results confirm and extend the observation that procaspase-3 expression in MCF-7 cells, which do not express spontaneously this protease, enhances the cell ability to undergo cell death in response to etoposide, methotrexate and other cytotoxic drugs [30]. Caspase-3 activation was confirmed by immunoblot showing the proteolytic cleavage of the protein. The cleavage of α-fodrin and lamin A, which was described as caspase-3 targets, also argues for a role of caspase-3 in these apoptotic pathways. In addition, siRNA-mediated down-regulation of caspase-3 in HBL100 decreased the apoptotic response to the drugs used, whereas caspase-3s expression inhibition increases cell death induced by the treatment in HBL100 and MDA-MB-231. It is important to note that there are no differences between HBL100 and MDA-MB-231 cells in expression of other apoptotic factor analyzed in this study. In MCF-7 cells, caspase-3 is absent and caspases-4 and -10 are downregulated. Nevertheless, as caspase-4 is an inflammatory caspase and caspase-10 is only involved in extrinsic apoptosis pathway, both these proteins have no influence on the studied apoptosis pathway.

In apoptosis involving the mitochondrial pathway, procaspase-3 is activated by caspase-9, subsequently to apoptosome formation [31]. Thus, it was of interest to precise the interaction between caspase-3s, pro-caspase-3 and/or caspase-9. Indeed, the ability of caspase-3s to interact with pro-caspase-3 and/or caspase-9 might, at least in part, contribute to explain its anti-apoptotic activity. We observed that procaspase-3 or caspase-3s expressed in MCF-7 cells interacted with active caspase-9 when these cells were exposed to apoptotic stimuli. This interaction was abrogated when caspase-3s and procaspase-3 are expressed simultaneously. These observations could suggest that interaction of active caspase-9 with a catalytically inactive caspase-3s could stimulate caspase-9 activity or activation at the apoptosome level explaining why, in MCF-7, the overexpression of caspase-3s alone increased slightly apoptosis rate. However this situation was observed only in MCF-7, which is deficient for caspase-3, and not in HBL100 as caspase-3s is expressed with procaspase-3 (Table S3). Nevertheless, in human tissues, caspase-3s is always expressed with procaspase-3. Taken together, these results strongly suggested that caspase-3s prevent the apoptosome assembly by sequestrating procaspase-3. These data evocate the mechanism of caspase-9 gene which also possesses a splice variant with antagonist apoptotic properties to the principal transcript. Indeed,, casp9-γ, an alternative splice variant of caspase-9, functions as an endogenous apoptotic inhibitor by interfering with the Apaf-1/procaspase-9 interaction [32]. Similarly, forced expression of the caspase-8 alternative splice variant, caspase-8L, protected hematopoietic cells from extrinsic apoptosis by preventing CD95 to connect to the caspase cascade [33].

In conclusion, our study indicates that caspase-3s could have its anti-apoptotic function by sequestration of procaspase-3, inhibiting the interaction of procasase-3 with caspase-9 and apoptosome, thus counteracting the activation of the apoptotic machinery (Figure 6). Our data support that the investigation of caspase-3s in breast tumors might contribute to explain certain forms of drug resistance, and to develop more adapted and efficient treatments.

**Figure 6:** Model of apoptosis inhibition by caspase-3s. After apoptotic signal, cytochrome c is released from mitochondria to the cytoplasm. Then, Apaf-1/cytochrome c oligomers are formed and interact with caspase-9. In presence of procaspase-3 only, the complex Apaf-1/cytochrome c/active caspase-9 interacts with procaspase-3 to form the complete apoptosome. Then, active caspase-3 is release from the complex and apoptosis occurs. In presence of caspase-3s, the complex Apaf-1/cytochrome c/active caspase-9 interacts with caspase-3s to form a “short” apoptosome having not the ability to induce apoptosis. Finally, in presence of both procaspase-3 and caspase-3s, caspase3s interacts with procaspase-3. This interaction induces the sequestration of procaspase-3, inhibiting the complete apoptosome assembly.

## Supporting Information

Figure S1 **Control of transfection by Western Blot assay with anti-GFP antibody in MCF-7 cell line.** Procaspase-3-GFP (ProC3-GFP) and caspase-3s-YFP (C3s-YFP) were stably overexpressed in single transfection and in co-transfection. GFP vector (GFP) was used as control. β-actin was used as loading control.
(TIF)

Figure S2 **Control of procaspase-3 and capsase-3s extinction after siRNA transfection.** **A.** Endogenous procaspase-3 was inactivated in HBL100 cells by siRNA transfection and the expression was monitored every 24 hours by western blot analysis from 24 to 96 hours after transfection. The transfection of siRNA induced the complete extinction of procaspase-3 from 48 to 96 hours after transfection. Caspase-3s expression was not affected by procaspase-3 siRNA transfection. **B.** Endogenous caspase-3s was inactivated in HBL100 and MDA-MB-231 cells by siRNA transfection and the expression was monitored every 24 hours up to 96 hours by real time quantitative PCR. The transfection of siRNA induced the complete extinction of caspase-3s from 48 to 96 hours after transfection. Nonetheless, procaspase-3 expression was not down-regulated by caspase-3s siRNA transfection, but its expression was strongly increased. **C.** The extinction of endogenous caspase-3s induced a strong increase of the endogenous procaspase-3/caspase-3s ratio. Double arrows indicate the optimal time lapse for cytotoxicity assay.
(TIF)

Table S1 Primers and probes sequences used in this study.
(DOC)

Table S2 Chemotherapeutic agents and doses used in this study to induce apoptosis.
(DOC)

Table S3 The cells (MCF7: deficient for caspase-3; HBL100: proficient for caspase-3) were incubated for 48 H in drug-containing medium and apoptosis was detected by flow cytometry. ^*^Data represent the percentage (± Standard Deviation) of apoptotic cells in each treatment conditions (mean of 3 experiments). CT: control, 5FU: 5- Fluorouracil, BLM: Bleomycine, CDDP: Cisplatin, EPI: Epirubicin, DOC: Docetaxol, VIN: Vincristine, STAU: Staurosporine. For the different drugs, the concentrations used to induce apoptosis are different in MCF-7 and HBL100, and are thus indicated in Table S2.
(DOC)

Table S4 Numbers indicate the mean fluorescence intensity of nuclei for each condition.
(DOC)
